# Malignant melanoma of the ileo-anal pouch anastomosis after restorative proctocolectomy for ulcerative colitis: report of a case

**DOI:** 10.1186/2047-783X-18-39

**Published:** 2013-11-04

**Authors:** Philipp Lingohr, Thomas Galetin, Hanno Matthaei, Eberhard Straub, Azin Jafari, Edwin Bölke, Jörg C Kalff, Karl-Heinz Vestweber

**Affiliations:** 1 Department of Surgery, University of Bonn, Sigmund-Freud-Strasse 25, Bonn 53127, Germany; 2 Department of Surgery, Klinikum Leverkusen, Am Gesundheitspark 11, Leverkusen 51375, Germany; 3 Department of Radiotherapy and Radiation Oncology, University of Düsseldorf, Moorenstrasse 5, Düsseldorf 40225, Germany

**Keywords:** Bowel, Malignant melanoma, Pouch, Ulcerative colitis

## Abstract

A 62 year-old patient with therapy-refractory pouchitis after proctocolectomy for ulcerative colitis was admitted with hematochezia and abdominal discomfort. A malignant melanoma (MM) was found after repeated biopsies of the pouch. Complete staging revealed no evidence for distant metastases and the patient underwent abdominoperineal pouch resection. Six weeks later, the patient was readmitted because of severe general deterioration and diffuse metastatic spread to the liver was found. The patient died of hepatorenal syndrome shortly thereafter.

Patients with inflammatory bowel disease are at increased risk of developing cancer, including rarities such as MM. Our experience stresses the importance of repeated biopsies in therapy-refractory pouchitis.

## Background

Inflammatory bowel diseases (IBD) are characterized by recurrent or chronic inflammation of the gastrointestinal tract mainly represented by Crohn´s disease and ulcerative colitis. Due to a very heterogeneous clinical presentations of patients affected and distinct courses of disease management of patients with IBD is challenging. Patients suffering from (IBD) are also at risk for developing cancer further complicating diagnostic and therapeutic decisions. We present a patient with ulcerative colitis who developed a malignant melanoma of the ileo-anal pouch anastomosis after restorative proctocolectomy.

## Case presentation

A 62 year-old man who had undergone proctocolectomy and ileal pouch anal anastomosis (IPAA) with a hand-sewn anastomosis for ulcerative colitis eight years previously developed pouchitis that did not respond to topical hydrocortisone (rectal foam) and oral prednisolone 20 mg/day. Prior representative biopsies from the inlet ileum and all thirds of the pouch had not revealed any malignant cells. Four months after the onset of his pouchitis symptoms, which were liquid stools combined with high frequency and incontinence resulting in a erosive dermatitis of the anal region, he was readmitted to our hospital complaining of pain in the anal region, meteorism, lower abdominal pain, diarrhea and loss of weight of about seven kilograms in four weeks.

Physical examination, ultrasonography, laboratory values, and hydro-magnetic resonance imaging (hydro-MRI) revealed no pathological findings except for leukocytosis (13.8 × 10^9^ cells/L). Pouchoscopy of the IPAA showed hemorrhagic and ulcerating pouchitis with stenosis of the proximal pouch (Figures 1 and 2). Biopsies showed both acute and chronic ulcerating inflammation with subtotal atrophy of the villi (Heidelberg Pouchitis Activity Score 10, scale 0 to 12, [1]). Surprisingly, we saw a circumscribed dark lesion in the proximal third of the pouch which we biopsied during a subsequent pouchoscopy. Immunohistochemistry confirmed a diagnosis of malignant melanoma (MM) (melan A positive, S100 and phosphoglucomutase-1 negative, Ki-67 positive in 80% of cells). We then performed thorough staging. A skin check by a dermatologist revealed two benign skin tumors (lentigo simplex and lentiginous compound nevus) that were completely excised. Examination by an otorhinolaryngologist and an esophagogastroduodenoscopy showed no abnormalities. Computed tomography of the thorax and abdomen and MRI of the pelvis showed enlarged regional lymph nodes and a partially thickened IPAA.

**Figure 1:** Pouchoscopy view showing ulcerative and hemorrhagic pouchitis with melanotic areas.

**Figure 2:** Pouchoscopy view showing stenosis of the ileal pouch anal anastomosis.

Two month after the initial presentation, the patient underwent complete resection of the pouch including the sphincter apparatus. Intraoperatively, the dorsal prostate gland was found to be adherent to the pouch close to the palpable mass. After consultation with our urologist colleagues, a tumor infiltration of the gland was strongly suspected and the prostate was resected *en bloc*. The patient recovered uneventfully from the procedure.

Histological examination of the pouch revealed ulcerated ileal mucosa and an invasive MM with atypical melanocytes invading the underlying submucosa. The lesion was composed of sheets of epithelioid melanocytes with melanin pigment that were positive for S100 and human melanoma black (HMB)-45 (Figures 3 and 4). Six resected mesenteric lymph nodes belonging to the pouch were infiltrated by the same cells but proved to respect the lymph node capsule.

**Figure 3:** Colonic mucosa with ulceration and foci of malignant melanoma containing atypical melanocytes invading the underlying submucosa (H&E, magnification × 16).

**Figure 4:** Invasive lesions composed of typical sheets of epithelioid melanocytes containing melanin pigment (H&E, magnification × 400).

Surprisingly, histological examination of the prostate revealed a synchronous adenocarcinoma (Gleason score 5 (2 + 3), TNM classification pT2, pNx, pMx, L0, V0, R0) although no infiltration by the MM could be evidenced.

In summary, the final diagnoses were MM of the anal mucosa with secondary infiltration of the ileal pouch after restorative proctocolectomy, and adenocarcinoma of the prostate.

All treatment decisions were strictly according to the recommendations of our weekly tumor board. After postoperative interdisciplinary discussion of this patient, close surveillance was recommended since there were no signs of distant metastases and, according to the literature, adjuvant therapy would have no proven benefit in this situation [2].

Six weeks after the patient was discharged from our hospital, he was readmitted because of further weight loss, lack of appetite and poor general health. Ultrasonography revealed diffuse metastatic spread to the liver. Multiple percutaneous biopsies taken under ultrasound control showed tumor cells that were negative for S100, slightly positive for HMB-45 and strongly positive for vimentin, confirming metastases from the previously diagnosed MM. We administered palliative chemotherapy with dacarbazine but the patient died of hepatorenal syndrome and subsequent multiorgan failure three weeks later.

## Discussion

Malignant melanomas of the intestinal tract are very rare. However, they account for 1 to 3% of malignant anal tumors [3], the anoderm being the third most common location for MM after the skin and retina. Yaramov *et al*. identified about 300 published reports of anorectal MM [4]. Because of its rarity, there are no prospective studies concerning anorectal MM. Thus, current knowledge is based largely on small uncontrolled retrospective series and lacks an evidence-based approach.

When we searched published reports for studies that included patients with primary MM of the intestinal tract, the largest series we found included 79 cases of anorectal MM [5], followed by one with 47 cases of rectal MM [6] and another with 19 cases of anorectal MM [7]. Poggi *et al*. reported 10 cases of colonic (not rectal) MM [8] and Elsayed *et al*. 103 patients with MM of the small intestine [9]. In addition, we identified several reports of single cases of small intestinal MMs that were predominantly located in the ileum [10]. Reports of esophageal MM demonstrate that such lesions can appear almost anywhere in the gastrointestinal tract [11-14].

Because MMs can arise in a great variety of locations and have a tendency to metastasize diffusely, determination of the primary site is a frequent challenge in their clinical management. Criteria that have been used for claiming the bowel as the primary site include absence of any evidence of skin or retinal MM, no identifiable metastases and, probably the most important, prolonged survival after R0 resection. Distinction between metastasis and primary tumor by histopathological examination is almost impossible [15].

Melanocytes originate in the ectoderm. Some histopathological studies hint at the possibility that anal melanocytes can migrate above the dentate line [16]; one report has described identification of melanocytes in the rectum [17]. During embryogenesis, melanocytes are believed to migrate to the ileal portion of the small intestine via the omphaloenteric duct [10]. Schwann cells and cells of the amine-precursor uptake and decarboxylation system are also thought to give rise to primary small intestinal MMs [18].

It is probable that the primary lesion is elsewhere in a majority of cases with claimed ‘primary bowel MM’. Since the overall five-year survival rate is only 10%, long-term survival after resection hints that the disease did indeed originate in, and was limited to, the bowel [19].

Radiation or chemotherapy do not seem to improve long-term survival. The only treatment from which patients can benefit is early and radical surgical resection before metastasis has occurred [2,18]. Cheung *et al*. used 1973 to 2004 data from the largest USA cancer registry to retrospectively study 659 cases of primary gastrointestinal melanoma [2]. Patients who underwent surgery had a significantly prolonged median survival time regardless of the degree of tumor differentiation and lymph node status, whereas radiation had no effect on median survival. Nonetheless, as is true of cutaneous melanoma, negative lymph nodes are a favorable prognostic factor, the median survival time after surgery being double that of patients with positive lymph nodes.

Patients with inflammatory bowel disease (IBD) such as Crohn’s disease and ulcerative colitis have an increased risk of non-melanotic skin cancer; this is probably attributable to light-sensitization caused by treatment with thiopurines [20]. They are also at increased risk of MM, probably because of immunosuppression by the IBD itself or treatment with immunosuppressive agents [21]. The association between colonic or small intestinal MM and IBD was first described 20 years ago [22]. Long *et al*. analyzed insurance data of about 100,000 patients with IBD and found a significantly increased risk of MM in patients with Crohn’s disease, but not in those with ulcerative colitis [23]. However, the risk of MM was increased in patients with both Crohn’s disease and ulcerative colitis who had undergone treatment with anti-tumor necrosis factor-alpha (TNF-α) antibodies. Anti-TNF-α antibodies have been increasingly used in severe cases of IBD over the last decade. TNF-α, a pro-inflammatory cytokine, is a pivotal mediator of IBDs. It triggers chemokine production, leading to leukocyte recruitment into the intestine and activating immune and endothelial cells and fibroblasts. Thus, it activates the immune system, including anti-tumor activity. TNF-α-blocking agents like infliximab induce apoptosis of immune cells, repressing inflammation in severe cases of IBD. Consequently, TNF-α blocking therapy increases the risk of infections and probably also of malignancies [24-26]. However, the absolute risk is small and does not negate the benefits of TNF-α inhibitors in severe Crohn’s disease [27]. Our patient had not received TNF-α inhibitors.

## Conclusion

Malignant melanoma of the intestinal tract is rare. To the best of our knowledge, this is the first reported case of a MM arising in the anal mucosa infiltrating an ileo-anal pouch. Our patient had no known risk factors for either this highly unusual tumor or his synchronous adenocarcinoma of the prostate. He did have hematochezia, lower abdominal pain and altered bowel habit, which are nonspecific but common symptoms in patients with bowel MM. His rapid tumor progression after surgery suggests that occult metastases may already have been present at the time of diagnosis. Thus, not all patients benefit from surgical treatment. Although postmortem studies reveal bowel metastases in 60% of patients with stage IV MM, intestinal metastases are diagnosed in less than 20% of patients with metastatic MM during life (reviewed in [15]).

In general, treatment should be based upon decisions by an interdisciplinary tumor board. Provided no metastases are found during staging, early surgical resection provides the only avenue for long-term survival in this disease [2].

We recommend repeated biopsies of the pouch in cases of pouchitis. Even if MMs are extremely rare lesions, other malignant tumors may occur on the backdrop of chronic inflammation. We particularly recommend biopsy sampling of all patients presenting with therapy-refractory pouchitis as presented here. In this situation, physicians should be aware of an increased risk for developing malignancies. In order to find evidence-based treatment algorithms whenever a malignant tumor is diagnosed, patients with rare entities should in the future be included in prospective randomized controlled trials.

## Consent

Written informed consent is available for review by the Editor-in-Chief of this journal.

## Abbreviations

H&E: Hematoxilin and eosin staining; IBD: Inflammatory bowel disease; IPAA: Ileal pouch anal anastomosis; MM: Malignant melanoma.

## Competing interests

Philipp Lingohr and the other co-authors have no conflicts of interest.

## Authors’ contributions

PL and TG: Evaluating the literature and the presented case. Writing the manuscript. HM, ES, AJ and EB: Writing parts of the manuscript and proofreading. JCK and KHV: Giving advice and proofreading of the manuscript. All authors read and approved the final manuscript.
